This article has been retracted.

# Clinical Study on Characteristics and Risk Factors of Coronary Artery Lesions in Young Patients with Acute Myocardial Infarction

**DOI:** 10.1155/2021/5716410

**Published:** 2021-10-04

**Authors:** Hua Liu, Jiangang Zhang, Zengcai Ma, Zesheng Xu

**Affiliations:** ^1^Tianjin Medical University, Tianjin, China; ^2^Department of Cardiology, Cangzhou Central Hospital of Tianjin Medical University, Tianjin, China

## Abstract

Epidemiological evidence suggests that the incidence of acute myocardial infarction (AMI) among people under 40 years of age has an increasing trend in recent years. Smoking, hypertension, diabetes mellitus, family history, and gender (male) are considered as classic risk factors for CHD, but the pathogenesis of CHD in young people is not exactly the same. Moreover, the relationship between the pattern of coronary artery disease and risk factors in young patients with acute myocardial infarction is inconclusive. In this study, we retrospectively studied the clinical data of 150 AMI patients treated in our hospital from January 2020 to May 2021. The patients were divided into the young group and elderly group according to the difference in age. The number of coronary artery lesions, the degree of coronary artery stenosis, the distribution dominance typing, the position of the lesions, and the presence of collateral circulation were observed and compared between the two groups. Multivariate logistic regression analysis was used to investigate the risk factors affecting coronary artery lesions in young patients with AMI. The results showed that the number of coronary lesions in young patients with AMI was mainly single-vessel, and the dominant type of distribution was mainly right dominant type. The stenosis degree is lighter than that of elderly patients, and the incidence of collateral circulation is lower than that of elderly patients, but the position of the lesions has no obvious regular. Smoking, staying up late, HDL-C, and LDL-C/ApoB were independent factors affecting the number of coronary artery lesions, and the changes of HDL-C and LDL-C/ApoB had an important influence on the degree of coronary stenosis in young patients. This provides a new idea for clinical treatment.

## 1. Introduction

AMI is a common cardiovascular disease, which not only affects the quality of life of patients but also brings heavy burden to society and family [1]. Because of its high mortality rate, it has become a serious threat to the global health and life safety of subpublic health problems [2]. With the development of social economy and the change of lifestyle, the incidence of AMI tends to be younger in recent years [3]. It is necessary to investigate the characteristics of coronary lesions and whether there are new risk factors or patterns of morbidity in young patients with myocardial infarction.

In 2018, a retrospective study of the clinical data of 360 AMI patients treated in Peking Union Medical College Hospital found that most AMI patients under the age of 30 were acute ST-segment elevation myocardial infarction, with single and nonobstructive lesions common, and the anterior descending branch was the most common criminal vessel [4]. This reveals the clinical and coronary artery lesion characteristics of patients with acute myocardial infarction under the age of 30. According to the lesions involved, single-vessel lesions, two-vessel lesions (including two-vessel lesions involving the left main artery), and three-vessel lesions are classified. Triple-vessel disease (TVD) is a serious type of coronary heart disease, namely, stenosis of right coronary artery, anterior descending artery, and circumrotatory artery. So, TVD has a higher incidence of cardiovascular events and mortality than single-vessel disease (SVD) and double-vessel disease (DVD) [5]. Dominant type refers to the main source of blood supply for the posterior descending branch of the heart and posterior collateral branch of left ventricle.

By retrieving the previous literature, we found that there were few domestic studies on the specific location of young AMI lesions and the relationship between thrombotic lesions and left and right coronary artery dominance [6]. In addition, the model relationship between coronary artery lesions and risk factors in young patients with acute myocardial infarction is still uncertain. Smoking and dyslipidemia are major risk factors for AMI, but the new research points out that high-risk occupations such as staying up late and dependence on electronic products may be new risk factors [7]. Based on this, this study analyzed the clinical data of 150 patients with AMI to explore the location and characteristics of coronary lesions in young patients with AMI during coronary angiography to analyze the relationship between coronary responsibility lesions and left and right coronary advantages, and to reveal possible new risk factors for the disease.

## 2. Materials and Methods

### 2.1. General Data

A retrospective study was performed on the clinical data of 150 patients with AMI who were admitted to our hospital from January 2020 to May 2021. Among them, 84 patients were younger than 45 years old and 66 patients were older than 60 years old and grouped as the youth group and elderly group, respectively. There were 47 males and 37 females in the youth group, with an average age of (38.84 ± 2.71) years old. There were 35 males and 31 females in the elderly group, with an average age of (69.16 ± 3.24) years old.

### 2.2. Inclusion Criteria

All patients met the third edition of the harmonized global definition of myocardial infarction published by the European Society of Cardiology (ESC) in 2018 [8]. Specifically, cardiac markers represented by troponin can be detected clinically at least once beyond the 99th percentile value of the upper limit of the normal reference value (URL) and accompanied by at least one of the following clinical indicators: accompanied by coronary artery blood supply caused by myocardial ischemia symptoms, new or possibly new significant ST-segment up or down or T-wave changes and new left bundle branch block (LBB), the presence of pathological Q-waves on ECG, and imaging examination found new myocardial loss or new segmental wall motion abnormalities. Clinical data were complete.

### 2.3. Exclusion Criteria

(i) Coronary artery and main branch vessel diameter stenosis <50%. (ii) Patients who had previously undergone coronary artery bypass grafting and/or prescriptive drug therapy. (iii) Patients who had normal coronary angiography results or (and) incomplete examination reports and imperfect medical records extraction. (iv) Women in pregnancy or lactation. (v) Patients with other cardiovascular and cerebrovascular diseases. (vi) Patients with dysfunction of other important organs. (vii) Mental illness or communication disorder.

### 2.4. Observation Method of Coronary Artery Lesion Characteristics

The right radial artery or right femoral artery was selected for puncture, and selective coronary angiography (CAG) was performed by the Judkins method. Generally, six projection positions are taken for the left coronary artery, including normal + head position 30°, normal + foot position 30°, left anterior oblique 30° + foot position 30°, left anterior oblique 30° + head position 30°, right anterior oblique 30° + foot position 30°, and right anterior oblique 30° + head position 30°. Three individual positions were taken for the right crown, including 45° left anterior oblique, 30° right anterior oblique, and 30° right anterior oblique + 30° head position. The projection postures can be increased in individual special cases according to the situation. The results of postoperative coronary angiography were judged by two experienced interventional physicians.

The characteristics of coronary artery lesions were described in the following ways. (i) The number of coronary artery lesions was divided into SVD, DVD, and TVD. (ii) The degree of coronary artery stenosis included four types: 50–75% for moderate stenosis, 76–90% for severe stenosis, 91–<100% for very severe stenosis, and 100% for complete occlusion. (iii) The distribution dominance typing included three types: left advantage type, right advantage type, and equilibrium type. (iv) The position of the lesions included four types: left main (LM), anterior descending branch (LAD), gyral branch (LCX), and right coronary artery (RCA). (v) The presence of collateral circulation was determined visually based on CAG images.

### 2.5. Data Collection and Methods

Literature and guidelines were reviewed; clinical data were collected through case review, analysis of coronary angiography images, and telephone follow-up. The risk factors included in this study included gender, family history of AMI, smoking history, and staying up late. At the same time, the laboratory test results of patients were recorded, including troponin, CK-MB, C-reactive protein, BNP, total cholesterol (TC), triglyceride (TG), high-density lipoprotein (HDL-C), and low-density lipoprotein (LDL-C)/apolipoprotein B (ApoB). Among them, the concept of staying up late is defined as not getting into sleep after 23:00 due to specific affairs (work, study, and games), voluntarily or involuntarily [9].

### 2.6. Statistical Methods

All data were processed with SPSS 22.0 statistical software, and GraphPad Prism 8 was used to make statistical graphs. Measurement data are expressed as mean ± standard deviation ($\bar{x}$ ± *s*), the independent sample *t*-test is used for comparison between groups, and analysis of variance (*F*) was used between multiple groups. Count data are expressed as (*n* (%)), and the chi-square (*χ*^2^) test is performed. Multivariate logistic regression analysis was used to study the risk factors of coronary artery disease in young patients with AMI. The difference is statistically significant when *P* < 0.05.

## 3. Results

### 3.1. The Number of Coronary Artery Lesions Was Compared between the Two Groups

The young group was mainly affected by single-vessel disease, while the elderly group was mainly affected by three-vessel disease. The number of cases of single-vessel disease and three-vessel disease between the two groups was statistically significant (*P* < 0.05, Table 1).

### 3.2. Comparison of the Degree of Coronary Stenosis between the Two Groups

The proportion of very severe stenosis and complete occlusion in the elderly group was higher than that in the young group, and the proportion of moderate stenosis and severe stenosis was lower than that in the young group, with a statistical significance (*P* < 0.05, Table 2).

### 3.3. Comparison of Distribution Advantages between the Two Groups

The distribution advantage types of the youth group and the elderly group were mainly right advantage type, and there was no statistical significance between the two groups (*P* > 0.05, Table 3).

### 3.4. Comparison of the Position of the Lesions and the Collateral Circulation between the Two Groups

LAD was the main position of the lesions in both groups, and there was no difference between the two groups (*P* > 0.05). The establishment of collateral circulation in the elderly group was higher than that in the young group, but there was no difference (*P* > 0.05, Table 4).

### 3.5. Regression Analysis of Risk Factors Related to the Number of Coronary Artery Lesions in the Young Group

The regression analysis was carried out with the number of lesions as dependent variables and gender, family history of AMI, history of smoking, troponin, CK-MB, C-reactive protein, BNP, TC, TG, HDL-C, staying up late, and LDL-C/ApoB as independent variables. The variable assignment is given in Table 5. 0.05 was the inclusion standard, and 0.10 was the exclusion standard. The fitting results showed that smoking, HDL-C, staying up late, and LDL-C/ApoB were the independent factors affecting the number of coronary artery lesions (*P* < 0.05). Young AMI patients with no smoking history, no HDL-C, staying up late, and abnormal LDL-C/ApoB had lower risk of multiple diseased coronary arteries (*P* < 0.05, Table 6).

### 3.6. Regression Analysis of Risk Factors Related to Coronary Artery Stenosis in the Young Group

The degree of coronary artery stenosis was used as the dependent variable, and gender, family history of AMI, history of smoking, staying up late, troponin, CK-MB, C-reactive protein, BNP, TC, TG, HDL-C, and LDL-C/ApoB were used as the independent variables for regression analysis. The variable assignment is given in Table 7. 0.05 was used as the inclusion standard, and 0.10 was used as the exclusion standard. The fitting results showed that staying up late, HDL-C, and LDL-C/ApoB were the independent factors affecting the severity of coronary artery stenosis in the young group (*P* < 0.05), and the risk of severe stenosis or complete occlusion was lower in young AMI patients without staying up late and abnormalities of HDL-C and LDL-C/ApoB (*P* < 0.05, Table 8).

## 4. Discussion

AMI is myocardial necrosis caused by acute and persistent ischemia and hypoxia of coronary artery. At present, there is no unified definition of young AMI. It is generally considered to be a heart disease caused by myocardial ischemia, hypoxia, and necrosis caused by acute occlusion of coronary arteries in adults younger than 45 years old [10]. According to epidemiological statistics, young AMI patients accounted for 3–10% of the total number of patients with coronary heart disease [11]. Coronary atherosclerosis is the primary cause of AMI. Studies have shown that coronary atherosclerosis can result in narrowing of the lumen of one or more coronary arteries and myocardial insufficiency [12]. On the basis of insufficient collateral circulation, fatigue, emotional excitement, stress response, and other inducements will lead to the rupture of unstable atherosclerotic plaques, the formation of lumen thrombosis, and the rupture of lumen. Once the blood supply decreases sharply, it will cause myocardial ischemia and develop into myocardial infarction. With the development of diagnosis and treatment methods for AMI, CAG has become the “gold standard” for the diagnosis of coronary heart disease [13]. Identifying the number of coronary lesions, coronary stenosis, location of coronary lesions, and the classification of dominant coronary arteries in young patients has important clinical significance for the individualized selection of reperfusion therapy [14].

Scholars have found that young patients with AMI have a high incidence of single-vessel coronary vascular disease, and most of them involve the anterior descending branch, and the necrotic myocardial area is smaller than that of the elderly [15]. Meanwhile, the atherosclerotic plaque in young patients is dominated by cellular fibrous tissue, which is often accompanied by intraplaque adipocytes and extracellular lipid accumulation, and a lower incidence of calcification. In this study, it was found through CAG that young patients mostly had single-branch lesions, generally involving the anterior descending branch, followed by the circumflex branch and the right coronary artery [16]. In contrast, the middle-aged and elderly patients had predominantly multibranch lesions with higher stenosis and establishment of collateral circulation than young patients. This clinical difference is basically consistent with previous studies, the cause of this clinical difference can be attributed to the fact that middle-aged and elderly patients are often accompanied by other complications, as well as their coronary vessels themselves calcification, weak elasticity, and low vascular endothelial function predispose them to acute thrombus formation [17].

Smoking is a traditional independent risk factor for coronary lesions in AMI. Previous studies have confirmed that nicotine in cigarettes can promote arterial wall smooth muscle recession and increase the platelet aggregation and thrombosis, inducing coronary artery spasm and causing AMI [18]. Besides, nicotine can also cause inflammatory reaction, massive secretion of various inflammatory mediators and matrix metalloproteinases in plaques, and increase the risk of plaque damage and ischemic events [19]. At the same time, according to the logistics regression model, staying up late was also an independent factor affecting the number of lesion branches and the degree of coronary artery stenosis [20]. This is because staying up late can cause sympathetic excitation, thus activating the renin-angiotensin system. The angiotensin not only has a strong proinflammatory effect but also can accelerate the rupture of plaques. It can also cause coronary artery contraction and thus reduce blood flow, which is not conducive to timely clearance of apoptotic bodies after macrophage apoptosis, and increases the risk of plaque thrombosis [21].

Abnormalities of lipid quality and quality are in HDL-C-reactive plasma. The LDL-C/ApoB can reflect the size of LDL particles, the horizontal state of B-type low-density lipoprotein particles, and the oxidative susceptibility of LDL particles and has the function of predicting the occurrence of cardiovascular disease [22]. Therefore, abnormal HDL-C and LDL-C/ApoB levels are closely related to hyperlipidemia. In this study, the data of patients diagnosed with AMI in our hospital were collected. The results of multiple logistics regression model analysis showed that HDL-C abnormality was an independent factor affecting the number of lesions and the degree of coronary artery stenosis. The relationship between dyslipidemia and atherosclerosis is clear, and the specific pathogenesis by which hyperlipidemia promotes atherogenesis includes two aspects. On the one hand, chronic hyperlipidemia (mainly hypercholesterolemia) can directly cause the endothelial cell dysfunction and increase the endothelial cell permeability [23]. On the other hand, hyperlipidemia can also increase the levels of oxidized LDL (ox LDL), which can and monocytes/macrophages combine to form macrophages to phagocytose lipids; meanwhile, chemotactic monocytes bind to endothelial cell adhesion molecules and stimulate various cytokines and growth factors production, finally forming atherosclerotic lesions [24].

In summary, the number of coronary lesions in young patients with AMI was mainly single-vessel, and the dominant type of distribution was mainly right dominant type. The stenosis degree is lighter than that of elderly patients, and the incidence of collateral circulation is lower than that of elderly patients, but the position of the lesions has no obvious regular. Smoking, staying up late, HDL-C, and LDL-C/ApoB were independent factors affecting the number of coronary artery lesions, and the changes of HDL-C and LDL-C/ApoB had an important influence on the degree of coronary stenosis in young patients. Early intervention on the above factors can achieve early prevention of young AMI and improve the prognosis of young AMI patients [25].

## Figures and Tables

**Table 1:** The number of coronary artery lesions was compared between the two groups.

Group	*n*	SVD	DVD	TVD
Young group	84	49 (58.33)	21 (5.00)	14 (16.67)
Elderly group	66	16 (24.24)	20 (30.30)	30 (45.45)
*χ* ^2^	—	17.493	0.523	14.777
*P*	—	≤0.001	0.469	≤0.001

**Table 2:** Comparison of the degree of coronary stenosis between the two groups.

Group	*n*	Moderate stenosis	Severe stenosis	Very severe stenosis	Complete occlusion
Young group	84	23 (27.38)	33 (39.29)	12 (14.29)	16 (19.05)
Elderly group	66	5 (7.58)	9 (13.64)	30 (45.45)	22 (33.33)
*t*	—	9.549	12.061	17.811	3.988
*P*	—	0.002	0.001	≤0.001	0.046

**Table 3:** Comparison of distribution advantages between the two groups.

Group	*n*	Left advantage type	Right advantage type	Equilibrium type
Young group	84	30 (35.71)	49 (58.33)	5 (5.95)
Elderly group	66	21 (31.82)	42 (63.64)	3 (4.55)
*t*	—	0.250	0.436	0.145
*P*	—	0.617	0.509	0.703

**Table 4:** Comparison of the position of the lesions and the collateral circulation between the two groups.

Group	*n*	The position of the lesions				The collateral circulation	
		LAD	LCX	RCA	LM	Yes	No
Young group	84	53 (63.10)	13 (15.47)	11 (13.10)	7 (8.33)	28 (33.33)	56 (66.67)
Elderly group	66	38 (57.58)	16 (24.24)	10 (15.15)	2 (3.03)	54 (81.82)	12 (18.18)
*t*	—	0.472	0.003	0.130	1.843	35.059	
*P*	—	0.492	0.956	0.719	0.175	≤0.001	

**Table 5:** Variable assignment table for risk factor analysis of the number to the coronary artery lesions in the youth group.

Variable	The assignment
Dependent variable	
The number of coronary artery lesions	SVD = 0, DVD = 1, TVD = 2

Independent variables	
Gender	Female = 0, male = 1
Family history of AMI	No = 0, yes = 1
History of smoking	No = 0, yes = 1
Troponin	Enter in actual value
Staying up late	No = 0, yes = 1
CK-MB	Enter in actual value
CRP	Enter in actual value
BNP	Enter in actual value
TC	Enter in actual value
TG	Enter in actual value
HDL-C	Enter in actual value
LDL-C/ApoB	Enter in actual value

**Table 6:** Regression analysis of risk factors related to the number of coronary artery lesions in the young group.

Independent variables	*b*_*j*_	SE (*b*_*j*_)	Wald *χ*^2^	*P*	95% CI	
					Upper limit	Lower limit
Gender	−0.540	0.236	2.165	0.571	−0.315	−0.046
Family history of AMI	−0.364	0.351	2.569	0.306	−0.569	−0.031
History of smoking	−0.461	0.245	6.792	0.026	−0.379	−0.146
Troponin	−0.548	0.104	12.536	≤0.001	−0.264	−0.012
Staying up late	−0.651	0.143	3.165	0.252	−0.462	−0.105
CK-MB	−0.547	0.105	3.758	0.164	−0.564	−0.131
CRP	−0.698	0.133	4.923	0.067	−0.262	−0.166
BNP	−0.518	0.126	5.109	0.059	−0.467	−0.261
TC	−0.694	0.108	4.789	0.074	−0.574	−0.365
TG	−0.733	0.135	5.341	0.055	−0.502	−0.243
HDL-C	−0.459	0.119	12.166	≤0.001	−0.475	−0.061
LDL-C/ApoB	−0.566	0.139	7.595	0.003	−0.316	−0.032

**Table 7:** Variable assignment table for risk factor analysis of coronary artery stenosis in the youth group.

Variable	The assignment
Dependent variable	
The degree of coronary artery stenosis	Moderate stenosis = 0; severe stenosis = 1; very severe stenosis = 2; complete occlusion = 4

Independent variables	
Gender	Female = 0, male = 1
Family history of AMI	No = 0, yes = 1
History of smoking	No = 0, yes = 1
Troponin	Enter in actual value
Staying up late	No = 0, Yes = 1
CK-MB	Enter in actual value
CRP	Enter in actual value
BNP	Enter in actual value
TC	Enter in actual value
TG	Enter in actual value
HDL-C	Enter in actual value
LDL-C/ApoB	Enter in actual value

**Table 8:** Regression analysis of risk factors related to coronary artery stenosis in the young group.

Independent variables	*b*_*j*_	SE (*b*_*j*_)	Wald *χ*^2^	*P*	95% CI	
					Upper limit	Lower limit
Gender	−0.621	0.216	5.085	0.252	−0.264	−0.103
Family history of AMI	−0.559	0.257	8.195	0.093	−0.361	−0.125
History of smoking	−0.425	0.341	10.674	0.068	−0.571	−0.266
Troponin	−0.433	0.285	10.526	0.075	−0.854	−0.285
Staying up late	−0.528	0.320	6.133	0.165	−0.369	−0.132
CK-MB	−0.643	0.169	6.587	0.149	−0.877	−0.344
CRP	−0.527	0.175	7.315	0.125	−0.633	−0.260
BNP	−0.396	0.147	8.527	0.088	−0.258	−0.105
TC	−0.451	0.188	10.988	0.063	−0.159	−0.155
TG	−0.533	0.392	9.507	0.079	−0.633	−0.138
HDL-C	−0.465	0.102	13.659	≤0.001	−0.532	−0.256
LDL-C/ApoB	−0.476	0.132	12.147	0.016	−0.285	−0.093

## Data Availability

The data used to support the findings of this study are available from the corresponding author upon request.
